# 3D Modeling of Sculpture Nano-Ceramics under Sparse Image Sequence

**DOI:** 10.1155/2022/5710535

**Published:** 2022-07-07

**Authors:** Zeyin Yang

**Affiliations:** Hefei Normal University, Hefei 230061, Anhui, China

## Abstract

To improve the analysis ability of point cloud 3D reconstruction of sparse images of nano-ceramic sculpture points, an automatic cloud 3D reconstruction method of nano-ceramic sculpture points based on sparse image sequence is proposed. Firstly, 3D angle detection and edge contour feature extraction methods are used to analyze 3D point cloud features of nano-ceramic sculpture point save image; secondly, the point cloud of the fuel economy image of nano-ceramic sculpture points is merged and the sloping action method is used to shape degradation to realize the information increase and fusion filtering of the fuel economy image of nano-ceramic sculpture points; finally, combined with the local mean denoising method, image is refined to improve the ability of sparse image outline structure of nano-ceramic sculpture points. The simulation results show that this method has high accuracy, good image matching ability, and high signal-to-noise ratio.

## 1. Introduction

With the development of 3D image processing technology, using 3D feature reconstruction and sparse scattered point structure reconstruction methods to extract and automatically reconstruct 3D features of sparse image sequences can improve the ability of automatic resolution and feature recognition of sparse image sequences. The three-dimensional reconstruction method of sparse image sequence is studied. The research of related image processing technology is of great significance in the fields of medical image processing, artificial intelligence recognition, and remote detection. In the process of sparse cloud image generation, the ability of automatic recognition of sparse points is improved. Using image information processing and analysis methods, energy-saving images of multilayer sculpture points are analyzed to improve the reconstruction and output detection capabilities of multilayered sculpture point-saving images. In traditional methods, the outline of the structure-saving technology of the fuel-based image sculpture mainly involves the following methods: RGB image structure method, block radon ruler structure method, point distribution model (PDM) method, and so on.

A conventional analysis method is used to reconstruct a saving image of sculptural dots to improve the resolution of the image, but this method has problems with excessive calculation cost and poor resolution. Aiming at the problems of traditional methods, an automatic three-dimensional construction method of a sculptural point cloud based on the energy-saving sequence is proposed. The 3D construction method, which is based on energy-efficient scatter points and sharpened template properties, is developed for 3D image construction, as shown in Figure 1.

## 2. Literature Review

3D reconstruction technology has attracted a lot of attention, and it is still a very active topic in academic research. The purpose of reconstruction is to restore the three-dimensional shape from the two-dimensional still images observed from different viewpoints. Many different research methods have been developed.

Kunii published the first batch of relevant research papers in the 1970s and called this method as SFS method [1]. Chen first proposed to restore the shape of the object from the brightness information of the image. The gradual change in the surface orientation of the space object causes the smooth change in the brightness of the image [2]. Hemami et al. combined the image illumination equation and smoothing constraint to form an objective function. Later, researchers successively introduced other methods to restore the shape of objects from two-dimensional images [3]. Krebs et al. introduced the integrability limit in the objective function [4]. Subudhi et al. proposed stereo photometry, fixing the position of camera and object, setting three light sources in different directions, and lighting in turn. Due to the limitation of integrability, the introduction of smooth limitation can be collectively referred to as the SFX method [5]. Remondino first proposed to determine the change in surface depth by texture or texture gradient in 1950 [6]. According to López-Aguirre et al., for the surface with mirror component, the method of four light sources is adopted to eliminate the influence in the calculation of variation line vector of mirror component [7]. Radicioni et al. proposed the photometric stereo method with two light sources. Although the photometric stereo method is easy to implement, it has some inevitable disadvantages: it is a point-by-point recovery method and is sensitive to noise [8]. Kim et al. believed that the principle of binocular imaging method is to use two cameras at different positions to shoot the object and observe the difference in the same point on the object in the two images [9]. Liu et al. believed that the camera baseline focal length can determine the spatial position of a point using a simple perspective relationship [10].

Based on current research, an automatic three-dimensional construction method of nano-ceramic sculpture points based on the energy-saving sequence is proposed. How to reconstruct a smooth sculpture model from sparse image sequence and reduce the number of images and workload has always been a problem of great concern. This study makes full use of two kinds of reliable and stable information in the image: occlusion contour and shadow. In this paper, the 3D reconstruction of sculpture is studied and three new geometric modeling methods are proposed.

## 3. Application of 3D Image in Nano-Ceramics of Sculpture under Sparse Image Sequence

### 3.1. 3D Image Reproduction Technology

#### 3.1.1. Introduction

This component realizes 3D image reproduction through the FDK algorithm. The FDK algorithm is a three-dimensional image structure algorithm proposed by Feldkamp and others. In the late 1970s, at present, most three-dimensional structure algorithms are extended based on this algorithm. The implementation rule for the FDK algorithm is presented below.  Figure 2 depicts the geometric coordinate relationship of a conical beam of a circular scanning path, where *O*-xyz represents the coordinate system of the world, *O*-uv represents the projection data coordinate system, and *O*-*x* represents the coordinate system of the radiator [11]. The *z*-axis is assumed to be the rotary station axis, and the s-axis always passes through the center of the radiator and is perpendicular to the aircraft sensor. For ease of analysis, this component of the sensor converts the projection data into the plane of the projection data passing through the source *O* according to the geometric scale, as shown in Figure 2.

FDK calculation mainly includes the following two steps, as shown in the following formulae:

(1) Filtering:
  (1) $$\begin{array}{c} P_{\theta }^{*}\left(i,j\right)=\left(\frac{d_{o}}{\sqrt{d_{o}^{2}+i^{2}+j^{2}}}P_{\theta }\left(i,j\right)\right)*h\left(i\right). \end{array}$$
(2) Back projection:
  (2) $$\begin{array}{c} f\left(x,y,z\right)=\int_{0}^{2n}u^{2}P_{\theta }^{*}\left(p,q\right)\text{d}\theta , \end{array}$$
  where dsO is used to describe the distance between the center of the ray source and the origin *O*; *Pθ* (*i*, *j*) and *P*^*∗*^*θ* (*i*, *j*) are used to describe the projection and filtered projection data under the rotation angle *o,* respectively; *h* (*i*) is used to describe the convolution function; (*P*, *q*) used to describe the back projection point address of the reconstructed volume on the projection plane; and *f* (*x*, *y*, *z*) is used to describe the reconstructed image data at voxel points (*x*, *y*, *z*). Assuming that the three-dimensional image of *N*3 size is reconstructed from *m* projected images, FDK is described by *C* language pseudocode according to equations (1) and (2).

#### 3.1.2. 3D Printing Platform System of Ceramic Products

3D printing technology can make the expression of ceramic product design stage more intuitive. Through 3D printing technology and 3D image reproduction technology, the overall shape of ceramic products can be reflected in an all-round and three-dimensional way [12]. Because the 3D printing technology is relatively flexible and the digital model has high operability and editability, the designer adjusts for new problems at any stage of design, and the time required to establish the digital model is significantly lower than that of manually drawing two-dimensional drawings and solid models. Because of the use of computer drawing, the efficiency is significantly improved and the effect is better. The 3D printing service platform system of ceramic products based on 3D image reproduction technology designed in this section is realized according to the characteristics of networked service platform. It mainly includes physical layer, service architecture layer, infrastructure layer, core application layer, and user layer. The architecture diagram is shown in Figure 3.

#### 3.1.3. Operation Mode of 3D Printing Service Platform for Ceramic Products

This section determines the operation mode of the 3D printing service platform of ceramic products according to the characteristics and requirements of 3D printing of ceramic products, combined with the supply form of 3D printing equipment resources of ceramic products, resource types, and user needs. Its overall framework and combination ideas are shown in Figure 4.

As can be seen from Figure 4, the designed platform provides a combination of pure online services and online and offline services. The types of services provided mainly include A, B, C, D, and E. In the 3D service platform for ceramic products, the resource provider, the resource demander, the platform service provider, and the platform operator share resources and participate in the platform together. The resource provider mainly provides ceramic design resources and manufacturing resources of 3D printing equipment; the resource demander is the user of 3D printing service platform for ceramic products; the platform service provider is mainly responsible for providing software technology, while the operator is mainly responsible for the use, maintenance, and management of the 3D printing service platform for ceramic products [13].

### 3.2. Reconstruction of 3D Model of Nano-Ceramic Sculpture from Occlusion Contour

Computer vision uses images to reconstruct geometry, and the simple and reliable method is based on shape from silhouette [14]. However, most of the existing occlusion contour methods are realized by volume intersection technology. In essence, the intersection of polyhedron is used to approximate the actual shape. When facing a smooth sculpture, a large number of pictures are required. On the one hand, it increases the amount of operation and calculation; on the other hand, we have to buy expensive electromechanical control systems. We analyze the constraints of occlusion contour and find that the volume intersection technology does not fully express the constraints. Therefore, a physical deformation technology is designed to fully realize the occlusion contour constraint through the repeated deformation process. Because the new method makes full use of the constraint information implicit in the image, it can reconstruct a better model from the same number of images; this is verified in an example.

#### 3.2.1. Occlusion Contour Constraint and Volume Intersection Technology

Due to the different light-reflecting properties of the object and the background, the contours of the closure line are formed during imaging, which limits the geometry of the object: the object must be located in the cone consisting of the perspective and the contours of the closure. [15]. When looking at different places, many cones are formed and the object must be located at the common intersection of these cones. Based on this concept, volume intersection technology is a mature method of restoring features from closed outlines. It directly uses the intersection of these cones as the approximation of the original object. However, volume intersection technology does not fully reflect the complete meaning of occlusion contour constraint. The resulting model is a conservative estimation of the actual shape and contains a large number of areas that do not belong to the interior of the object. The line of sight passing through the occluded contour not only limits the boundary of the object, but also is tangent to the surface; occlusion contour constraints are touch constraints, not cut constraints. Fully expressing this constraint, we should get better reconstruction results. Therefore, we design a new method to realize the above idea, which mainly includes three steps. Firstly, the traditional volume intersection processing is carried out using the occlusion contour to obtain the triangular mesh model; then, the simplified mesh model is transformed into the triangular Bezier surface model; finally, through physical deformation technology, the shape of Bezier surface is adjusted to fully meet the occlusion contour constraints [16].

#### 3.2.2. Smooth Bezier Surface Generation

In previous work, we have implemented volume intersection technology to obtain the dense triangular mesh model. To facilitate the later deformation operation, the envelope algorithm is used to simplify the model, and a smooth quadric Bezier surface model is constructed on the simplified model. Because the topology of the object surface is unknown in advance, only triangular Bezier patches suitable for any structure type can be used to interpolate the simplified mesh vertices and maintain the cross-boundary tangent vector continuity between patches. Shadow is another kind of easily processed information in the image. The shadow produced on the surface of an object due to its own unevenness is called self-occlusion shadow; when an object is located between a plane and the light source, it can produce a projection on the plane, which is equivalent to the area surrounded by the occlusion contour observed in the direction of the light source, which is called silhouette. An improved method in this chapter is to use silhouette to extract occlusion contour quickly and reliably, to realize 3D reconstruction based on occlusion contour; at the same time, with the help of the shadow of the object surface, the cutoff contact position between the light blocking the contour and the object surface can be obtained [17]. Compared with the method in the previous chapter, using the known contact information to optimize the surface model is not only more efficient but also more accurate. In addition, this section also analyzes the imaging change law of self-occlusion shadow on the object surface during the rotation of the object and its shape constraints on the concave area and puts forward another reconstruction method that can deal with the concave shape.

### 3.3. Nano-Ceramics

#### 3.3.1. Characteristics and Types of Nano-Ceramic Materials

Nano-oxide powder is a metastable intermediate material with nano-size (1 ∼ 100 nm) between solid and molecule. Nano-ceramic powder materials have the following excellent properties:

1. Nano-ceramic materials have very small particle size, large specific surface area, and high chemical activity, which can reduce sintering sealing temperature and save energy. It is usually 400 ∼ 600°C lower than engineering ceramics, and there is no need to add any sintering additives. It densifies and homogenizes the composition and structure of the material, improves the performance of the ceramic material, and improves its reliability.
2. The composition and structure of nano-materials can be controlled from the structural level (1 ∼ 100 nm), which is conducive to give full play to the potential properties of ceramic materials and make the directional design of microstructure and properties of nano-materials possible.
3. Because ceramics are sintered after processing and forming of raw materials, and the particle size of ceramic powder determines the microstructure and macro properties of ceramic materials, if the particles of the powder are evenly stacked, the sintering shrinkage is consistent and the grains grow evenly, the smaller the particles, the fewer defects, and the higher the strength of the prepared materials.

## 4. Using Silhouette Shadow Information to Reconstruct 3D Model of Complex Body

### 4.1. Spline Surface Reconstruction Using Silhouette Information

The object is placed on the rotating platform, the high-intensity parallel light source is used for lateral illumination, and a plate is placed in the vertical irradiation direction to make the object produce a clear silhouette on it. The camera takes images of objects and their silhouettes at the same time. Before taking the rotating image sequence of the object, first a cuboid is used as the calibration object to adjust the position and direction of the direct light source so that the light is perpendicular to the surface of the plate; then, the traditional method is used to calibrate the camera. The silhouette can be extracted by a simple idle value segmentation algorithm to obtain the occlusion contour; the image of an object can also be divided into light and dark areas [18]. According to the previous calibration information, each point on the occlusion contour can correspond to a light perpendicular to the plate, which “touches” the object surface, and the traditional volume intersection method can be realized by these lights. Using the projection matrix of the camera, the occluded contour light is first re-projected back to the image, and the image intersects with the image of the object. In the intersecting public section, the first light and shade dividing point in the reverse direction of light are the image of the intersection of line of sight and light, and its spatial position coordinates can be obtained by calculating the shortest distance between two straight lines. This point is actually the contour generation point, which is the tangent contact between the light and the object surface. Compared with the existing methods based on occlusion contour, it is not only easy to extract occlusion contour but also provides additional contact information of line and surface. In this way, the spline surface reconstruction method can be improved directly. The new method is improved, and the whole process is also divided into three steps: firstly, the initial 3D model is reconstructed by volume intersection technology, and the spatial mesh is formed by MC algorithm; then, the mesh is simplified and a smooth spline surface model is constructed; finally, the spline model is optimized using the “touch” meaning of occlusion contour constraint. The methods of the first two steps are the same, but the last optimization step is improved. In the previous section, there is a large amount of calculation in spline surface optimization. On the one hand, in the “tensioning” step, the shortest distance is found between lines and surfaces. First, the patch is found by searching where the nearest distance point is located, and then the nearest distance point is determined by finding the minimum value [19]. When the exact position of the cutting contact is unknown, it needs to be solved iteratively from multiple initial points many times. In addition, the shortest distance point obtained is not necessarily near the real cutting contact. Therefore, it needs repeated “tension” and “relaxation” steps to stabilize. Under the imaging system in this section, the cutoff contact information has been obtained, and the shortest distance between line and surface has been transformed into the shortest distance between point and surface, which greatly reduces the amount of calculation, and it can be stabilized without multiple “tension” and “relaxation” steps, which further reduces the amount of calculation, as shown in Figure 5.

### 4.2. Reconstruct the Shape of the Depression Area from the Self-Occlusion Shadow

The efficiency and accuracy of 3D reconstruction based on occlusion contour are greatly improved using a light-dark boundary on the object surface, but it still cannot deal with the concave area. Between the light and shade dividing line corresponding to the cutting contact and the light source, there are other self-shading shadows on the object surface, which reflect the depression of the object surface. In the imaging system of this section, the surface of the rotating platform is horizontal and the rotating axis is perpendicular to the horizontal plane. The shape of the object can also be described by the profile on each horizontal plane. We consider the constraint of self-occlusion shadow on the horizontal profile, as shown in Figure 6.

#### 4.2.1. Comparison of Several Different Reconstruction Methods

When calculating the cutting contact, the light generated by the occlusion contour has been re-projected back to the image. Although this light no longer intersects with the object surface between the cutting contact and the light source, its re-projection is regarded as the section between the corresponding light plane and the object surface, and the error will not be great. Moreover, for the convenience of discussion, it is assumed that the camera adopts parallel projection and the line of sight direction is perpendicular to the light direction. When considering the cross-sectional profile, the problem is simplified to the ZD case. The following illustration shows the different characteristics of the traditional method. In the traditional method, the contact constraint that blocks the contour line of the object is actually simplified to the cutting constraint. In other words, the object must be in a convex polygon as shown in the diagram, but whether the object has a tangential relationship to the polygon, and where the tangential points are, no consideration was given.

#### 4.2.2. Reconstruction of Concave Area from Self-Occlusion Shadow

The real contact information is used, but the depression area cannot be processed; this section reconstructs the depression with self-occlusion shadows. Self-occlusion shadow has two constraints on the shape of the profile [20]. One is the contact constraint, and the other is the visibility constraint. As shown in the figure, a shadow generated by a light source with illumination direction *L* is observed in the direction of line of sight *v*. One of all rays is tangent to the surface to generate the observed shadow, which is called shadow generation line. Generally, only the shadow generation line is known to be in the parallel band formed by scanning the shadow segment along the observation direction. When the position of the shadow generation line is known, a tangent constraint is formed on the surface shape of the object: the shadow generation line has two points be corresponding to the shadow segment along the light direction, be must be on the object surface, and the tangent of the surface at point B is the shadow generation line. In addition, the point of view of the object contained in EB cannot move to any scanning direction. The shape of the depression area will be inferred from these two constraints. Each ray direction (i.e., the direction of the shadow generation line) is exactly parallel to each edge of the surrounding polygon, which provides convenience for storing shadow information [21]. The position information of the shaded segment on each horizontal section can be stored on the edge of the surrounding polygon. It should be noted that the shadow segment is not necessarily completely within each side, but may be on its extension line. This method of storing the shadow segment information on the edge of the surrounding polygon does not mean that the shadow area corresponding to the object surface is on the corresponding edge. The shadow of each segment is extended along the observation direction and cut into the surrounding polygon, the cutting contact (on the surrounding polygon) is taken as the boundary, and the polygon is re-segmented (i.e., the adjacent cutting contact is marked as the same segment, which is composed of the straight edge after two segments are cut) [22]. It can be proved that each shadow segment must be projected within the boundary of a certain segment, and any cutting contact cannot fall into any shadow segment. In this way, the shadows can be classified according to the projection position of each shadow segment on the surrounding polygon. Those located in the same boundary interval are the same category, and their shadow areas will be on the same boundary segment [23–25].

## 5. Conclusion

This study mainly studies the 3D modeling method of complex sculpture body based on sparse image sequence and its application. How to reconstruct a smooth sculpture body model from sparse image sequence and reduce the number of images and workload has always been a problem of great concern. This study makes full use of two kinds of reliable and stable information in the image: occlusion contour and shadow, studies the 3D reconstruction of sculpture, and puts forward three new geometric modeling methods of sculpture.

1. Firstly, starting with the analysis of occlusion contour constraints, the initial 3D model is reconstructed by volume intersection technology, and the spatial mesh is formed by the MC algorithm; then, the mesh is simplified and a smooth spline surface model is constructed; finally, the spline module is optimized using the “touch” meaning of occlusion contour constraint. The first two shortcomings of occlusion contour information are solved; that is, the number of images required is reduced, and a more smooth object surface can be obtained.
2. In view of the difficult problem of occlusion contour extraction and the large amount of calculation in the previous method, a simple imaging system is designed, which not only simplifies the occlusion contour extraction but also uses the point information generated by the silhouette to extract the occlusion contour quickly and reliably, so as to realize the 3D reconstruction based on the occlusion contour. At the same time, with the help of the shadow of the object surface, the cut contact position between the light passing through the occlusion contour and the object surface can be obtained.
3. Finally, under the same imaging system, the shape restriction of the self-occlusion shadow on the object surface on the concave area is studied, and the relevant constraints are obtained. Therefore, a simple concave area reconstruction method is realized, which makes it possible for the simple passive vision method to reconstruct the non-convex complex shape.
4. These algorithms are programmed with MATLAB language. The passive computer vision system is difficult to realize the reconstruction of depression area. Based on the previous research and analysis, this study solves this deficiency. The methods in this study are innovative. The simulation of these methods through programming makes these methods possible to be practical. Due to time constraints, these methods still have some shortcomings. In the future work, we should still focus on reducing the number of images needed for reconstruction and smoothing the reconstruction results. The research shows that this method requires less a priori knowledge, shorter time overhead, and less error.

## Figures and Tables

**Figure 1:** Automatic 3D reconstruction of sculpture point cloud.

**Figure 2:** Geometric coordinate relationship of cone-beam pattern scanning track.

**Figure 3:** 3D printing platform system of ceramic products.

**Figure 4:** 3D platform operation mode.

**Figure 5:** Surface reconstruction of silhouette information.

**Figure 6:** Constraint of self-occlusion shadow on horizontal profile.

## Data Availability

The data used to support the findings of this study are available from the corresponding author upon request.
